# LINC00461 Regulates the Recurrence of Large B Cell Lymphoma through the miR-411-5p/BNIP3 Pathway

**DOI:** 10.1155/2022/9100056

**Published:** 2022-06-24

**Authors:** Shu-wen Sun, Yan Chen, Hui-juan Liao, Wei Zhang, Wen-ming Xu, Guo-qian He

**Affiliations:** ^1^Key Laboratory of Birth Defects and Related Diseases of Women and Children, Ministry of Education, West China Second University Hospital, Sichuan University, Chengdu, Sichuan 610041, China; ^2^Department of Pediatrics, West China Second University Hospital, Sichuan University, Chengdu, Sichuan 610041, China; ^3^Joint Laboratory of Reproductive Medicine, Key Laboratory of Birth Defects and Related Diseases of Women and Children, West China Second University Hospital, Sichuan University, Chengdu, Sichuan 610041, China; ^4^Department of Medical Oncology, Sichuan Cancer Hospital & Institute, Sichuan Cancer Center, Cancer Hospital Affiliate to School of Medicine, Chengdu, Sichuan 610041, China

## Abstract

**Objective:**

To analyze the mechanism of LINC00461 regulating the recurrence of diffuse large B cell lymphoma (DLBCL) through microRNA (miR)-411-5p/BCL2 interacting protein 3 (BNIP3) pathway.

**Methods:**

DLBCL samples in TCGA and GSE12453 were used for differential analysis to find long noncoding RNA (lncRNA) related to DLBCL recurrence. The 4 DLBCL data with the highest and lowest expression levels of LINC00461 in the TCGA database were selected for GSEA enrichment analysis. The targeting relationships of miR-411-5p with LINC00461 and BNIP3 were verified by the dual luciferase report. Blood samples from DLBCL patients were used to analyze the correlation between miR-411-5p and LINC00461 or BNIP3. LINC00461, miR-411-5p, or BNIP3 was overexpressed or silenced by transfection, and a tumor-bearing nude mice model was constructed to detect their effects on proliferation and apoptosis.

**Results:**

The level of LINC00461 in DLBCL was significantly higher than that in normal cases, and the level in recurrence DLBCL was significantly higher than that in nonrecurrence. The enrichment analysis results showed that the function of LINC00461 was closely related to apoptosis. The results shown that miR-411-5p bound to LINC00461 and BNIP3 and was negatively correlated with LINC00461 and BNIP3 mRNA in blood of DLBCL patients. Suppressing the level of LINC00461 inhibited cell proliferation and induced apoptosis. The inhibition of LINC00461 or overexpression of miR-411-5p reduced the expression of BNIP3 protein, thereby inducing apoptosis at the in vivo and in vitro levels.

**Conclusion:**

LINC00461 may induce miR-411-5p to “sponge,” thereby increasing the expression of BNIP3 protein, and exerting the function of inhibiting apoptosis and promoting DLBCL recurrence.

## 1. Introduction

Diffuse large B cell lymphoma (DLBCL) accounts for about one-third of all lymphomas [1,2]. DLBCL clinically mainly manifests as painless progressive lymphadenopathy or local masses, or accompanied by fever and other organ or system symptoms [3]. The prognosis of different DLBCL patients is quite different. Among them, the 5-year overall survival rate of GCB-type DLBCL patients is 76%, while the 5-year overall survival rate of non-GCB-type DLBCL patients is only 34% [4]. Recurrence is an important factor in the death of DLBCL patients [5–7]. Analyzing the molecular mechanism of recurrence is of great significance for prognostic judgment and new drug development.

The regulatory mechanism of noncoding RNA (ncRNA) after transcription is a new focus of research. MicroRNA (miRNA) is a type of short (contains about 22 nucleotides), conserved endogenous RNA [8]. They efficiently bind to the 3′-untranslated region (UTR) of message RNA (mRNA). This kind of complementary base pairing can prevent translation or induce mRNA degradation [9]. When miRNA is “sponged” by the long noncoding RNA (lncRNA), the functions of the miRNA are inhibited, and the expression level of the target gene increases. The role of lncRNA-miRNA in DLBCL is gradually revealed. For example, lncRNA SMAD5-AS1 eventually increases the expression of APC by sponging miR-135b-5p and thus plays a role in inhibiting the proliferation of DLBCL cells [10]. lncRNA SNHG8 inhibits the level of miR-335-5p and inhibits the apoptosis of DLBCL cells through competitive endogenous RNA (ceRNA) [11]. However, the amount of lncRNA is huge. With the help of gene chip and bioinformatics analysis methods, we can comprehensively analyze the level of the transcriptome to find the key lncRNA [12,13].

In this study, we compared and obtained the differential genes between normal lymphoid tissues and DLBCL tissues, as well as the differential genes between recurrence and nonrecurrence DLBCL tissues. lncRNA LINC00461 was obtained. Enrichment analysis was used to find key genes downstream of LINC00461 to construct ceRNA regulatory pathways. The effects and mechanism of LINC00461 on DLBCL were analyzed through in vivo and in vitro experiments.

## 2. Materials and Methods

### 2.1. Bioinformatics Methods

In order to analyze the lncRNA related to the recurrence of DLBCL, the data in TCGA were downloaded, and a total of 3 recurrence patients and 3 nonrecurrence patients were obtained with clear indication. To compare the expression of lncRNA in DLBCL tissues and normal tissues, GSE12453 in the GEO database was selected, which included 5 cases of normal and 5 cases of DLBCL. The differences were analyzed separately, and the edgeR package in the R language was applied. The difference conditions were log|FC|>1, *P* < 0.05. The top 10 according to log|FC| were listed. The common lncRNA LINC00461 among the two differential genes was singled out.

To analyze the function of LINC00461, in the TCGA database, according to the expression level of LINC00461, the highest and lowest 4 cases were selected. Enrichment analysis was performed by gene set enrichment analysis (GSEA) via GSEA software 3.0, Massachusetts Institute of Technology, and Regents of the University of California.

### 2.2. Cells Culture and Treatment

Human DLBCL cell lines, OCI-Ly7, GM12878, FARAGE, U2932, and TMD8, were maintained in the DMEM complete medium containing 10% fetal bovine serum (FBS), 100 mg of streptomycin/mL, and 100 units of penicillin/mL (Solarbio, Beijing, China). The cells were cultured in a 5% CO_2_ incubator at 37°C and 95% humidity.

To analyze the influence of LINC00461, miR-411-5p, and BNIP3 on the biological behavior of DLBCL cells, the pcDNA3.1 carried human full-length LINC00461, siLINC00461, BNIP3, miR-411-5p mimic, and corresponding negative control (NC) plasmids were from GenePharma (Shanghai, China). After the cells in the 6-well plate reached 60%, Opti (100 *μ*L, Invitrogen, Waltham, USA) and Lipofectamine^TM^ 2000 (5 *μ*L, Invitrogen, Waltham, USA) were added and incubated for 5 min (A). Opti (100 *μ*L), pcDNA3.1 DNA (20 ng/*μ*L), mimic, or NC were added and incubated for 5 min (B). A and B were mixed and incubated for 20 min. After 16 h, the medium was changed, and the cells were harvested for subsequent experiments.

### 2.3. RT-qPCR

Briefly, total RNA in cells was extracted by TRIzol reagent (Thermo Fisher Scientific, Waltham, MA, USA). For LINC00461, using the PrimeScript RT reagent kit (Takara, Shiga, Japan), each total RNA sample (1 *μ*g) was subjected to reverse transcription reaction to obtain the cDNA template. The qPCR amplification was executed with SYBR Green reagent (Takara, Tokyo, Japan) using the ABI 7500 fast real-time PCR system (Applied Biosystems, Foster City, CA, USA) with the following conditions: 95°C for 10 s, followed by 40 cycles of 95°C for 10 s, 50°C for 30 s, and 72°C for 30 s. The expressions of lncRNA and mRNA were normalized to GAPDH using the 2^−ΔΔCt^ method.

For miR-411-5p, total miRNA was extracted using miRNeasy Mini kit (GE Healthcare, USA), and cDNA was formed by TaqMan miRNA reverse transcription kit (DBI Bioscience, Germany). Then, the TaqMan miRNA kit (DBI Bioscience, Germany) was applied to measure the expression level of miRNA. The expression of miRNA was normalized to U6 using 2^−ΔΔCt^ method.

The sequences were as follows: miR-411-5p mimic, 5′-UAGUAG ACCGUAUAGCGUACG-3′; miR-411-5p inhibitor, 5′-CGU ACGCUAUACGGUCUACUA-3′; LINC00461: forward (5′-3′) GACATTTACGCCACAACCCACG; reverse (5′-3′): AGACAGACCCTCAGATTCCCCA. U6: forward (5′-3′) CTCGCTTCGGCAGCACA; reverse (5′-3′) AACGCTTCACGAATTTGCGT.

### 2.4. Western Blot

The cells were incubated with RIPA lysis solution on ice for 30 min. Cell lysate samples were centrifuged for 20 min at 4°C, 1500 × *g* to obtain the supernatant. The concentration of total proteins in the supernatant was determined using BCA kit (Beyotime Biotechnology, Jiangsu, China). In addition, proteins were separated using an Ambion PARIS^TM^ Kit (Invitrogen, Carlsbad, CA, USA) strictly according to the instructions. SDS-PAGE was applied for the separation of proteins. After being transferred to a polyvinylidene fluoride (PVDF) membrane (EMD Millipore, USA), proteins were blocked with 5% skimmed milk for 2 h at room temperature. Rabbit anti-BNIP3 (1:1000, ab109362, Abcam, Cambridge, MA, USA) was then added onto the membrane to incubate proteins overnight at 4°C. Thereafter, Tris-buffered saline/0.1% Tween (TBST) solution was used to wash the membrane twice. Horseradish peroxidase-labeled goat anti-rabbit IgG secondary antibody (1 : 2000, ab6721) was used to incubate the membrane for 2 h at 37°C. Thrice washing with TBST was performed on the membrane. The protein blots were visualized using enhanced chemiluminescence (ECL) (Solarbio, China), and image analysis software IPP6.0 was applied for the analysis of gray intensity. GAPDH was served as the internal control.

### 2.5. CCK-8 Assay

100 *μ*L of cell suspension was added into wells of 96-well plates with 5 replicate wells. After 48 h, CCK-8 solution with a volume of 10 *μ*L was added into each well to incubate cells for 2 h. At 450 nm wavelength, the optical density (OD) value of each well was detected with a microplate reader (Biotek, Winooski, VT, USA).

### 2.6. Acridine Orange/Ethidium Bromide (AO/EB) Staining

A glass cover slip was preplaced in a 6-well plate to make cell slide. The cells were fixed with 95% ethanol at room temperature for 15 min. 100 mg/L of AO (Sigma, St.Louis, MO) dissolved in PBS and 100 mg/L of EB (Sigma, St.Louis, MO) dissolved in PBS were mixed, each with 5 *μ*L, and then immediately added to the cells. After 30 s, it was observed using a confocal laser microscope (LSCM880NLO, Zeiss, Germany).

### 2.7. Flow Cytometry

For apoptosis, cells were washed with 1 × PBS and suspended in 100 *μ*L binding buffer. 5 *μ*L Annexin V-FITC and 10 *μ*l PI (Yeasen, Shanghai, China) were added and incubated in dark for 10∼15 min at room temperature. In the last, 400 *μ*L 1 × binding buffer was added into the sample and detected the sample by flow cytometry (Becton, NY, USA) within 1 h.

### 2.8. Dual Luciferase Report

The 3′-UTR sequence of wild-type (wt-) BNIP3 mRNA was amplified to the downstream site of the pGL4 luciferase vector (Promega, Madison, WI, USA). The rapid site-directed mutagenesis kit (D0206, Beyotime, Shanghai, China) was used to generate the mutated (mut-) BNIP3 mRNA 3′-UTR. The TMD8 cells were seeded in 24-well plates at a density of 3 × 10^4^/well. After 24 h, 1 *μ*g of wt-BNIP3 mRNA 3′-UTR or mut-BNIP3 mRNA 3′-UTR luciferase plasmid, 50 nM miR-411-5p mimic or miR-411-5p NC, and 150 ng of Renilla luciferase plasmid (Beyotime, Shanghai, China) were transfected into cells via Lipofectamine^TM^ 2000. The cells were then incubated at 37°C for 36 h. According to the manufacturer's protocol, a dual luciferase reporter gene detection kit (Promega, Madison, WI, USA) was used to detect luciferase activity. All data were normalized to Renilla luciferase activity. For the verification of the targeted binding of LINC0461 and miR-411-5p, the method was like the above description.

### 2.9. Animal Study

Nude mice (Slac Laboratory Animal Company, Shanghai, China) used for xenograft were divided into 3 groups: NC, BNIP3, and BNIP3 + shLINC00461. According to the groups, the transfected TMD8 cells were suspended with PBS in the density of 5 × 10^6^ cells, and 100 *μ*L suspension was injected subcutaneously into the left armpit area of the mice. After 28 d, the mice were euthanized by cervical dislocation. During the experiment, the pain of the mice was reduced as much as possible without affecting the results. This study was approved by the Animal Care and Use Committee of West China Second University Hospital, Sichuan University.

### 2.10. Immunohistochemistry

The tumor tissue samples were dehydrated with a gradient concentration of ethanol (70%, 4°C, 2 h; 80%, 4°C, 2 h; 90%, 4°C, 2 h; 100%, 4°C, 2 h; 100%, 4°C, 2 h). Then, the samples were immersed in paraffin (<60°C, 2 h), and after embedding in paraffin, the section thickness was 5 microns. Xylene was used for dewaxing, and then, the samples were treated with various levels of ethanol and finally washed with distilled water.

### 2.11. Blood Samples

From January 2015 to January 2016, 65 DLBCL patients were collected. These patients were all diagnosed with DLBCL and had not received relevant antitumor therapy before enrollment. These 11 patients were 35-74 years old, 34 males and 31 females. Peripheral blood samples of these patients were collected. The levels of LINC00461, miR-411-5p, and BNIP3 mRNA were detected by RT-qPCR. All patients were informed and agreed. This study was approved by the ethics committee of Sichuan Cancer Hospital.

### 2.12. Statistical Analysis

All experiments were performed independently three times. Data were presented as mean ± standard deviation (SD) and were processed by SPSS19.0 software (SPSS Inc., Chicago, IL, USA). Student's *t*-test was used for the comparison between two groups. For the comparison among at least three groups, one-way analysis of variance (ANOVA) was applied. The Pearson test was used to analyze the correlation between miR-411-5p and LINC00461 and BNIP3. *P* < 0.05 indicated that the difference was statistically significant.

## 3. Results

### 3.1. LINC00461 Is Upregulated in DLBCL and Is Associated with Recurrence

DLBCL data of 3 cases of recurrence and 3 cases of nonrecurrence in TCGA were analyzed for difference, and the results were displayed in heat map and volcano map (Figures 1(a) and 1(c)). According to the value of log|FC|, the top 10 lncRNAs are shown in Figure 1(e). In GSE12453, the difference analysis results between normal tissue and DLBCL tissue are shown in Figures 1(b) and 1(d), and the top 10 lncRNAs are shown in Figure 1(f). Among them, LINC00461 existed in the results of the two (Figures 1(g) and 1(h)). This suggested that LINC00461 was overexpressed in DLBCL and might be involved in tumor recurrence.

### 3.2. LINC00461 Participates in the Progression of DLBCL by Regulating Apoptosis

In order to further analyze the function of LINC00461, the 4 cases with the highest and lowest expression of LINC00461 were selected for GSEA enrichment analysis (Figure 2(a)). The results showed that the function of LINC00461 had the highest correlation with apoptosis (the *P* value was the smallest, Figure 2(b)). Based on this, we conducted in vitro experiments. Firstly, the expressions of LINC00461 in human DLBCL cell lines OCI-Ly7, GM12878, FARAGE, U2932, and TMD8 were detected by RT-qPCR. The results showed that LINC00461 was the highest in TMD8 cells (Figure 2(c)). Then, we used three types of siLINC00461 for transfection and found that they could significantly reduce the level of LINC00461 in cells (Figure 2(d)). The two groups with the largest decrease were selected for subsequent biological behavior research. The results of CCK-8 experiment showed that when the level of LINC00461 was reduced, and the proliferation activity of cells was significantly reduced (Figure 2(e)). AO/EB staining and flow cytometry were applied to detect apoptosis. As shown in Figure 2(f), it could be clearly seen from the picture that after LINC00461 was inhibited, the red fluorescence representing apoptosis increased. The results of flow cytometry also showed that inhibiting the expression of LINC00461 significantly induced the apoptosis of DLBCL cells (Figure 2(g)). In this part, we found that the function of LINC00461 was enriched in the apoptosis pathway through GSEA enrichment analysis. The cell experiment results also showed that inhibiting LINC00461 promoted apoptosis. This suggested that LINC00461 might promote the recurrence of DLBCL by inhibiting apoptosis.

### 3.3. LINC00461 Increases Bcl-2 Interacting Protein 3 (BNIP3) Protein Expression by Targeting miR-411-5p

To analyze the molecular mechanism of LINC00461 regulating DLBCL cell apoptosis, based on the principle of ceRNA, the corresponding miRNA was obtained using blast in the NCBI database, and then, the downstream target gene BNIP3 was obtained through online databases (https://targetscan.org, https://mirdb.org, https://microRNA.org). The binding sites of miR-411-5p and LINC00461 and BNIP3 are shown in Figure 3(a). LINC00461 and siLINC00461 were transfected with TMD8 cells to overexpress and inhibit LINC00461. The results showed that the overexpression of LINC00461 caused a decrease in the expression of miR-411-5p and an increase in the expression of BNIP3 protein in the cells. The inhibition of LINC00461 increased the level of miR-411-5p and reduced the expression of BNIP3 protein (Figures 3(b), 3(c), 3(f)). In addition, inhibiting miR-411-5p increased the level of BNIP3 protein in TMD8 cells. The overexpression of miR-411-5p not only inhibited the level of BNIP3 protein in TMD8 cells, but also blocked the promotion of BNIP3 protein by overexpression of LINC00461 (Figures 3(d)–3(f)). The results of the dual luciferase report experiment also confirmed that miR-411-5p could target LINC00461 and BNIP3 mRNA (Figure 3(g)). In order to further analyze the relationship between LINC00461/miR-411-5p/BNIP3 at the clinical level, the expression of LINC00461, miR-411-5p, and BNIP3 mRNA in 65 cases of DLBCL was detected by RT-qPCR. The results showed that miR-411-5p was negatively correlated with LINC00461 and BNIP3 mRNA, respectively (Figure 3(h)). This suggested that LINC00461 might increase BNIP3 protein expression by targeting miR-411-5p, thereby participating in the progression of DLBCL.

### 3.4. The Proproliferation and Antiapoptotic Functions of BNIP3 Are Targeted and Regulated by LINC00461/miR-411-5p

To further verify that LINC00461/miR-411-5p participated in the proliferation and apoptosis of DLBCL cells by regulating BNIP3, TMD8 cells were divided into 4 groups: NC, BNIP3, BNIP3 + siLINC00461, and BNIP3 + mimic. The results showed that the inhibition of LINC00461 and the overexpression of miR-411-5p could reduce the expression of BNIP3 protein (Figures 4(a) and 4(b)). The results of the CCK-8 experiment showed that the overexpression of BNIP3 increased cell viability, while the cell viabilities of the BNIP3 + siLINC00461 group and the BNIP3 + mimic group were significantly lower than that of the BNIP3 group (Figure 4(c)). The results of apoptosis-related experiments also showed that the overexpression of BNIP3 inhibited the apoptosis of TMD8 cells. The apoptosis rates of the BNIP3 + siLINC00461 group and the BNIP3 + mimic group were significantly higher than those of the BNIP3 group (Figures 4(d) and 4(e)). It was shown that the cancer-promoting effects of BNIP3 were reduced by the inhibition of LINC00461 and the overexpression of miR-411-5p. This further suggested that LINC00461 might promote the expression of BNIP3 by sponging miR-411-5p, thereby inhibiting DLBCL cell apoptosis.

### 3.5. LINC00461 Promotes BNIP3 and Induces the Progression of DLBCL

To further analyze that LINC00461/BNIP3 regulated apoptosis and promotes DLBCL on the in vivo level, the above four groups of cells were injected subcutaneously to construct tumor-bearing nude mouse model. The results showed that the overexpression of BNIP3 significantly increased tumor volume and quality. The inhibition of LINC00461 and BNIP3 alleviated the cancer-promoting effects of BNIP3 (Figures 5(a) and 5(b)). Through immunohistochemical staining, it was showed that in tumor tissues, the increase of BNIP3 promoted the expression of Ki67 and Bcl-2 protein, and inhibited Bax protein. The inhibition of LINC00461 reduced the expression of BNIP3 protein in tumor tissues, but also inhibited Ki67 and Bcl-2, and increased the level of Bax protein (Figure 5(c)). These experimental results confirmed in vivo that LINC00461 might increase the level of BNIP3 protein to promote Ki67 and Bcl-2 expression, but inhibit Bax, thereby inducing cell proliferation and reducing apoptosis.

## 4. Discussion

The first-line treatment for DLBCL is rituximab + CHOP, and recurrence is still an important factor in patient death [14,15]. In this study, in order to find the lncRNA related to DLBCL recurrence, the transcriptome information in DLBCL and normal tissues is compared, as well as the transcriptome information in recurrence and nonrecurrence DLBCL. The results show that LINC00461 is a differential gene, and its level in DLBCL is significantly higher than that in the normal group. In addition, the level of LINC00461 in recurrence DLBCL is also significantly higher than that in the nonrecurrence group. LINC00461 has a cancer-promoting effect in a variety of tumors, including colorectal cancer [16], breast cancer [17], lung cancer [18], gastric cancer [19], and so on, and in vitro experiments confirm that LINC00461 can promote tumor cell proliferation, migration, invasion, or inhibit apoptosis. In rectal cancer [20] and breast cancer [21], LINC00461 also promotes the resistance of tumor cells to cisplatin and docetaxel. However, there are almost no reports on LINC00461 and DLBCL or lymphoma. Based on this, it is preliminarily speculated that LINC00461 may participate in the promotion of DLBCL recurrence, and LINC00461 is the object of this study.

To analyze the function of LINC00461 in DLBCL, the 4 DLBCL data with the highest and lowest expression levels of LINC00461 in the TCGA database are selected for GSEA enrichment analysis. The results show that the function of LINC00461 is most enriched in the apoptosis pathway. It is showed that LINC00461 is elevated in multiple myeloma, and LINC00461 promotes the expression of Bcl-2 protein by targeting miR-15a/miR-16, thereby inhibiting cell apoptosis [22]. The inhibition of LINC00461 reduces the expression of antiapoptotic protein Bcl-2 by increasing the expression of miR-195, thereby promoting apoptosis and increasing the sensitivity of lung adenocarcinoma cells to radiation [23]. In gastric cancer, LINC00461 also plays an antiapoptotic effect [19]. Accordingly, this study mainly analyzes the effect of LINC00461 on DLBCL cell apoptosis. The results show that inhibiting the expression of LINC00461 reduces cell viability and significantly induces apoptosis. This preliminarily suggests that LINC00461 may participate in the occurrence and recurrence of DLBCL by inhibiting apoptosis.

To further analyze the antiapoptotic mechanism of LINC00461, the downstream miRNA and apoptosis-related target genes are predicted. The results show that LINC00461 can target miR-411-5p and regulate the expression of BNIP3 protein. miR-411-5p is found in lung cancer [24], oral squamous cell carcinoma [25], and renal cell cancer [26] and can inhibit tumors by promoting apoptosis. lncRNA SNHG15 can spongy miR-411-5p through the target and increase the expression of VASP protein, thereby inhibiting cell apoptosis [27]. BNIP3 is a protein that interacts with the antiapoptotic protein Bcl-2, and it is showed that BNIP3 drives the migration and invasion of melanoma cells and promotes angiogenesis by regulating integrin-related proteins [28,29]. BNIP3 is high in endometrial cancer tissues, and high levels of BNIP3 are related to postoperative adverse reactions, suggesting that BNIP3 is involved in recurrence [30]. However, it is showed that the loss of BNIP3 is involved in tumor proliferation and lymphatic metastasis [31]. It is found by Chen [32] that miR-145 inhibits the proliferation of prostate cancer cells and promotes apoptosis by targeting the expression of BNIP3 protein, thereby inhibiting tumor progression. The results of this study in vivo and in vitro show that the overexpression of BNIP3 can promote the proliferation of DLBCL cells, promote tumor growth, and inhibit cell apoptosis, increase the level of Bcl-2, and reduce Bax. Silencing LINC00461 and overexpression of miR-411-5p both inhibited the expression of BNIP3 and blocked the antiapoptotic and cancer-promoting effects of BNIP3. This further suggests that LINC00461 may increase the expression of BNIP3 protein, promoting Bcl-2 and inhibiting Bax, thereby inhibiting cell apoptosis, and participating in the progression and recurrence of DLBCL.

In summary, LINC00461 may be related to the recurrence of DLBCL. LINC00461 can increase the expression of BNIP3 protein by targeting miR-411-5p, thereby inhibiting the apoptosis of DLBCL. This suggests that LINC00461 may become a biomarker for predicting the prognosis of DLBCL and a new target for the treatment of DLBCL.

## Figures and Tables

**Figure 1:** LINC00461 is upregulated in DLBCL and is associated with recurrence. (a) Heatmap of the difference analysis between recurrence and nonrecurrence DLBCL in the TCGA database. (b) Heatmap of the difference analysis of GSE12453 (normal vs. DLBCL). (c) Volcano map of the difference analysis between recurrence and nonrecurrence DLBCL in the TCGA database. (d) Volcano map of the difference analysis of GSE12453 (normal vs. DLBCL). (e) The results of the difference analysis between recurrence and nonrecurrence DLBCL in the TCGA, according to the multiple of the difference, and the top 10 items were listed. (f) The results of the difference analysis of GSE12453, according to the multiple of the difference, and the top 10 items were listed. (g) Comparison of LINC00461 expression in recurrence and nonrecurrence DLBCL. (h) Comparison of LINC00461 expression in normal and DLBCL. ^*∗*^*P* < 0.05 vs. nonrecurrence or normal.

**Figure 2:** LINC00461 participates in the progression of DLBCL by regulating apoptosis. (a)-(b) GSEA enrichment analysis between the 4 cases of DLBCL data with the highest and lowest LINC00461 in TCGA. (c) The expression levels of LINC00461 in DLBCL cells. (d) LINC00461 expressions in TMD8 cells after transfection with different siLINC00461. (e) The effects of reducing the expression level of LINC00461 on cell viability. (f) Apoptosis detected via AO/EB staining; 200×. (g) Apoptosis detected via flow cytometry. ^*∗*^*P* < 0.05 vs. NC.

**Figure 3:** LINC00461 increases Bcl-2 interacting protein 3 (BNIP3) protein expression by targeting miR-411-5p. (a) The binding sites of miR-411-5p with LINC00461 and BNIP3. (b) The expression levels of miR-411-5p in TMD8 cells of each group. (c–f) The expression levels of BNIP3 protein in TMD8 cells of each group. (g) The dual luciferase report was used to verify the targeted binding of miR-411-5p to LINC00461 and BNIP3. (h) Correlation between miR-411-5p and LINC00461 and BNIP3. ^*∗*^*P* < 0.05.

**Figure 4:** The proproliferation and antiapoptotic functions of BNIP3 are targeted and regulated by LINC00461/miR-411-5p. (a)-(b) The expression levels of BNIP3 protein in TMD8 cells of each group. (c) Comparison of cell viability of different groups. (d) Comparison of apoptosis of different groups via AO/EB staining; 200×. (e) Comparison of apoptosis of different groups via flow cytometry. ^*∗*^*P* < 0.05.

**Figure 5:** LINC00461 promotes BNIP3 by sponging miR-411-5p and induces the progression of DLBCL. (a) Comparison of tumor volume of tumor-bearing nude mouse models in each group. (b) Comparison of tumor quality of tumor-bearing nude mouse models in each group. (c) Comparison of Ki67, BNIP3, Bax, and Bcl-2 protein expression levels in tumor tissues of each group; 200×. ^*∗*^*P* < 0.05.

## Data Availability

The datasets analyzed during the current study are available from the corresponding author upon request.
